# Effect of Precision Health Education on Compliance Behavior after Extracorporeal Shock Wave Lithotripsy

**DOI:** 10.1155/2022/3306036

**Published:** 2022-09-14

**Authors:** Chan-can Li, Zong-wu Zhang

**Affiliations:** Department of Urology, Anhui No.2 Provincial People's Hospital, Hefei, Anhui 230041, China

## Abstract

**Objective:**

The aim of this study was to investigate the effects of precision health education on patients' compliance behavior and lithotripsy efficacy after extracorporeal shock wave lithotripsy (ESWL).

**Methods:**

From June 2018 to September 2018, 104 patients with upper urinary tract calculi who underwent ESWL at Anhui No.2 Provincial People's Hospital were randomly divided into two groups. The observation group (*n* = 53) was given precision health education guidance after ESWL treatment, while the control group (*n* = 51) was only informed of precautions after lithotripsy. Postoperative compliance behavior, stone expulsion time, and complications were recorded in both groups.

**Results:**

The clinical baseline data of the two groups were similar in age, gender, number of stones, size of stones, location of stones, complications, number of lithotripsies, and voltage of lithotripsy between the two groups (*P* > 0.05). However, compared with the control group, the observation group had better compliance behavior of patients. Furthermore, we divided the patients into three groups based on whether they complied with medical advice. Compared with the noncompliance group (*n* = 17) and the partial compliance group (*n* = 23), the stone expulsion time in the complete compliance group (*n* = 64) was significantly shorter. Also, the number of patients with nausea and vomiting, lacrimation, and cold sweat in the complete compliance group was significantly lower than that in the other groups.

**Conclusion:**

Precision health education for patients treated with ESWL can significantly enhance the compliance behavior of patients, thereby accelerating the expulsion of stones, improving the efficacy and relieving pain. Precision health education and good compliance behavior complement and reinforce each other.

## 1. Introduction

Urolithiasis is an important source of morbidity worldwide and is a common urinary system disorder [1]. Due to changes in diet and lifestyle, its prevalence has increased by 10.6% and 7.1% in male and female patients, respectively [2]. Patients with urolithiasis often experience clinical symptoms such as abdominal pain and dysuria, which seriously impact the patient's life [3]. Despite the numerous treatments available for urolithiasis, the disease tends to recur after treatment and has a 10-year recurrence rate as high as 50% [4].

Extracorporeal shock wave lithotripsy (ESWL) is a noninvasive technique emerging in the 1980s for treating most stones, with the advantages of high safety, high efficacy, low pain, and rapid recovery. In addition, ESWL is easily accepted by patients and can be performed in the outpatient clinic. However, the stone-free rate after lithotripsy still needs to be improved, and a lack of appropriate postoperative management may result in serious complications such as hydronephrosis and infection, increasing the patient's pain to varying degrees [5, 6]. As an attempt to solve these issues, Zhang and Lu [7] recommended precision health education after ESWL, a personalized diagnosis and treatment model for stone expulsion, which was proven to significantly improve the stone-free rate after ESWL for urinary calculi and reduce the risk of postoperative complications.

However, the impact of precision health education on patients' compliance has not yet been studied. Thus, this paper collected the data of 104 patients with upper urinary tract calculi (UUTC) who underwent ESWL from June 2018 to September 2018 at the Anhui No.2 Provincial People's Hospital. They were divided into two groups (with or without precise health education after ESWL), and the patients' compliance, therapeutic effects, and complications were compared. This study was designed with the aim that the obtained results would provide a reference for the application of precise health education after ESWL for urolithiasis to improve patients' outcomes.

## 2. Materials and Methods

### 2.1. Study Subjects

Information on UUTC patients treated in the Department of Urology at the Anhui No.2 Provincial People's Hospital from June 2018 to September 2018 was retrieved and analyzed. The study inclusion criteria were as follows: (1) diagnosed with UUTC by X-ray, kidney, ureter, and bladder (KUB) X-ray/intravenous urography (IVU) or B ultrasound examination; (2) the clinical symptoms were characterized by lumbar and abdominal pain, hematuria, urinary urgency, and frequency; (3) absence of urinary tract infection and had a normal renal function; and (4) voluntarily signed the informed consent. Exclusion criteria were as follows: (1) age < 18 years; (2) combined urinary tract infection and renal insufficiency; and (3) had a previous history of ESWL or surgery for UUTC on the affected side. Eligible patients were then randomly divided into a control group (*n* = 51) and an observation group (*n* = 53). This study was approved by the Ethics Committee of Anhui No.2 Provincial People's Hospital (2022-0112).

### 2.2. Clinical Baseline Data of Patients

We collected the following clinical baseline data of patients: age, gender, education level, occupation, number of stones, size of stones, location of stones, comorbidities, number of lithotripsy, voltage of lithotripsy, and number of shocks.

### 2.3. Procedures of Extracorporeal Shock Wave Lithotripsy (ESWL)

The medical staff inquired about the detailed past medical history of the patients. In particular, elderly patients received careful measurement of blood pressure, pulse, and electrocardiogram before treatment to identify possible preventable anomalies during treatment. Then, the medical staff patiently explained the relevant knowledge of lithotripsy treatment and precautions to the patients and relatives and tried to alleviate negative psychological reactions such as anxiety, which helped the patients to cooperate with the treatment procedures. An imported dual-positioning Dornier lithotripter was used to complete the operation at a voltage of 12–14.5 kV. The procedure was started with 12 kV low energy for 100–500 shocks, and the power was gradually increased. In total, no more than 4000 shock waves were delivered. The whole process of ESWL was operated by one person and monitored. ESWL time was recorded, with an interval between two treatments of no less than 7 days. Patients or their family members gave informed consent and cooperated with the treatment.

### 2.4. Precision Health Education after Treatment

Precision health education [7] was given to the observation group immediately after ESWL, and the specific guidance is shown in Table 1. In contrast, for patients in the control group, only general precautions were introduced after lithotripsy, with no specific requirements and conventional health education. All patients were followed up for 3 months and reexamined by B ultrasound or KUB every 1 to 2 weeks to assess the compliance behavior and lithotripsy effects.

### 2.5. Observation Measures

Time of stone expulsion after the operation was observed. The criteria for successful stone expulsion were as follows [8]: After the patient felt that the stone was discharged, B ultrasound and KUB detected no stone in the patients or only detected shatters of diameter ≤ 3 mm in patients without clinical symptoms. Failure to expel stones was described as follows: after 1 month of ESWL, stone shadows could still be observed by B ultrasound or X-ray, and residual stones > 3 mm or require other surgical adjuvant therapy.

The compliance behavior of patients was graded as complete, partial, or nil based on the following: (1) *complete compliance*: patients completely followed the health education provided by doctors after ESWL, and all the items were implemented; (2) *partial compliance*: patients partially followed the health education after ESWL and performed items they considered important but ignored items they believed unimportant; (3) *noncompliance*: patients refused to receive the health education after ESWL and ignored all the treatment items.

Postoperative complications, such as hematuria, infection, lumbar soreness, nausea and vomiting, frowning, lacrimation, and cold sweat, were recorded and analyzed.

### 2.6. Statistical Analysis

The experimental data were statistically analyzed using the SPSS 17.0 software. Enumeration data were expressed as *n* (%), and chi-square (*χ*^2^) test or Fisher's exact test was used for comparison between groups. Measurement data were expressed as mean ± standard deviation (SD), and *t*-test was used for comparison between two groups. Univariate analysis was performed for comparison between multiple groups. *P* < 0.05 was used as the criterion for judging statistically significant differences.

## 3. Results

### 3.1. Patients' Baseline Clinical Data

In this study, 104 patients with UUTC aged 20-70 (median age: 41) years old were selected as the study subjects, including 73 males and 31 females. There were 8 cases of renal calculi, 64 cases of upper ureteral calculi, 13 cases of middle ureteral calculi, 19 cases of lower ureteral calculi, and 2 cases of distal ureteral calculi. No significant difference was observed between the control and observation groups in age, gender, number of stones, size of stones, location of stones, comorbidity, number of lithotripsy, and voltage of lithotripsy (*P* > 0.05), except for education level (*P* = 0.044), occupation (*P* = 0.002), and number of shocks (*P* = 0.025) (Table 2). Among the initially collected 104 cases, 2 patients in the control group lost contact because of going abroad.

### 3.2. Comparison of Compliance Behavior between the Two Groups

In this study, the compliance of patients in the two groups was analyzed (Table 3). The results showed that the compliance behavior of patients in the observation group was significantly better than those in the control group (*P* < 0.01), suggesting that precision health education guidance helped improve patients' postoperative compliance behavior.

### 3.3. Comparison of Stone Expulsion Time

We divided the patients into 3 groups based on whether they complied with medical advice. The results showed that the stone expulsion time in the complete compliance group was significantly shorter than that in the other two groups, and the time was longest in the noncompliance group (*P* < 0.05) (Table 4).

### 3.4. Comparison of Postoperative Pain Behavior

We compared the postoperative pain behavior of patients in the three groups. The results of Table 5 show that the number of patients who developed nausea and vomiting, lacrimation, and cold sweat postoperatively was significantly lower in the complete compliance group than in the other two groups (*P* < 0.05). However, there was no significant difference in the number of patients with lumbar soreness and frowning between the three groups (*P* > 0.05).

## 4. Discussion

Patient compliance represents patients' behavior in the prevention, treatment, and rehabilitation of diseases consistent with medical advice [9]. During medical treatment, the degree of compliance behavior of patients might be directly related to the stone expulsion rate after ESWL and the prevention of complications. In turn, a reduction in ESWL efficacy affects the confidence and satisfaction of patients with treatment, thereby reducing their compliance behavior. Collectively, compliance behavior and treatment outcomes show a close relationship.

Disease cognition is a prerequisite and guarantee for reducing symptoms, controlling the condition, and improving quality of life [10]. Active participation is vital to increasing disease cognition, but before participation, a good and specific self-management model for patients during follow-up after ESWL must be established. Some patients have little knowledge of ESWL or are unwilling to abide by recommendations, leading to low compliance toward medical orders after ESWL, failure to follow medical guidance, and interruption of postoperative follow-up, which consequently affect their treatment outcomes. As a result, about one-third of patients experience serious postoperative complications due to the remaining small pieces of stones [5, 11]. Some patients even believe that after all stones have been broken down by lithotripsy, there should be no stones remaining, and the recurrence of renal colic triggers a tense doctor-patient relationship. Some patients have good disease cognition but still refuse to follow the postoperative management; even with their families' participation, encouragement, or supervision, they reluctantly follow the doctor's advice. Thus, these are the common preventable issues that affect patients' compliance behavior after ESWL, thus making precision health education essential for patients with stones.

In addition, considering that conventional health education provides no comprehensive understanding of patients' psychological needs, changes in their condition, and individualized measures conducive to the effect of postoperative stone expulsion [7], thus, timely and effective “personalized” adjustment to post-ESWL management cannot be achieved [7]. Comparatively, precision health education after ESWL can provide personalized and optimal guidance for stone expulsion treatment. Specifically, based on the full understanding of the psychological needs of patients after ESWL, medical staff can establish personalized guidance for postural movement, self-management of stone expulsion, and adjuvant medication and other measures for each individual. Importantly, this guidance takes into account the characteristics of stones, the urinary tract environment where stones are located, and the patients' general condition. Several studies have shown that precision health education after ESWL can effectively improve SFR after ESWL and reduce the risk of postoperative complications, which is worthy of clinical application and promotion [7].

The primary need of patients after ESWL is stone expulsion. Precision health education can make ESWL achieve its best therapeutic effect and enable the tangible and invisible, immediate, and whole-course expression of feelings between doctors and patients, thus improving patient compliance. Residual stones are relatively common after ESWL, and although the ureter has peristaltic functions that promotes the passing of small stone pieces, more attention should be paid to residual fragments < 5 mm. It has been reported that residual stones < 5 mm can grow in 21% to 59% of patients after ESWL [12]. With the implementation of stone expulsion management guided by precision health education after ESWL, the recurrence of stones after surgery can be reduced. For stones that cannot be successfully expelled by conventional health education guidance after ESWL, the expected lithotripsy effect can be achieved through a personalized model of stone expulsion diagnosis and treatment if patients have high compliance with medical orders. According to our results, the observation group receiving precision health education was superior to the control group in patient compliance. Furthermore, we divided the patients into 3 groups (complete compliance, partial compliance, and noncompliance groups) according to whether they complied with medical advice or not. Compared with the noncompliance group and the partial compliance group, the stone expulsion time in the complete compliance group was significantly shorter. Also, the number of patients with nausea and vomiting, lacrimation, and cold sweat in the complete compliance group was significantly lower. These findings confirm that precision health education can improve patients' compliance after ESWL, which in turn can lead to effective lithotripsy and reduce patients' postoperative pain behavior.

Studies have shown compliant patients' behaviors are closely related to their personalities and psychological characteristics [13]. Thus, medical staff should meticulously explain and provide individualized precision health education and other active care services to positively affect patients' compliance and treatment outcomes. By analyzing the collected data, we found that precision health education after ESWL had the following advantages: (1) improve medical staff and patient relationships by making the patients fully understand the importance of postoperative follow-up and reexamination, (2) provide a platform to properly inform patients about the possible postoperative complications and provide psychological counseling to relieve patients' postoperative tension and anxiety, and (3) provide personalized guidance of precision health education according to the different stone sites. Thus, adequate humanistic care and timely communication between doctors and patients improve continuous stone expulsion treatment in patients after ESWL and reduce the risk of postoperative complications.

Further, we found that the two groups of patients had no severe hematuria and steinstrasse (or stone street) after surgery, possibly due to the small size of most stones and adequate preoperative preparation. For instance, anti-infection therapy was performed first if patients had an infection before lithotripsy so that no severe infection would occur after surgery in the two groups. Low contributor severity improves patients' compliance, thereby enhancing treatment efficacy.

In conclusion, precision health education after ESWL represents an individualized optimal management program for the treatment of stone expulsion and follow-up according to the location and size of stones, lithotripsy effect, and postoperative symptoms of patients. It has been shown to significantly improve the compliance behavior of patients, thereby accelerating stone expulsion, improving the efficacy of treatment, and relieving pain. Thus, these findings indicate that precision health education and good compliance behavior complement and reinforce each other.

## Figures and Tables

**Table 1:** Precision health education program after extracorporeal shock wave lithotripsy.

Item	Main content
Issue *patient reexamination form*	Explain the significance of follow-up; inform follow-up time and contact number.

Water intake and frequency	Inform postoperative water intake and frequency of the specific physical condition of patients. Generally, more than 2.5–3 L/d of water, equally distributed throughout the day, is recommended. In particular, patients are recommended to drink water before bedtime, after meals, and at night and maintain a urine volume of >2000 mL. Patients with renal colic attacks were recommended not to increase water intake during the day.

Postoperative medication guidance	Inform on the dose, usage, and adverse reactions of postoperative drugs. Patients with emergency ESWL and postoperative renal colic should stop taking drugs for stone expulsion on the same day but only receive routine antibacterial drugs.

Postoperative postural movement	After treatment, patients drink 500 to 1000 mL of water first, and postural movement is performed 10 to 15 min later. Postoperative movement is limited to 1–2 days according to individual differences in physical condition and stone expulsion progress. Different postural movements correspond to stones at different locations. *Stones situated in the upper calyx, middle calyx, renal pelvis, and ureter*: upright jumping (such as rope skipping and step jumping) with the heel landing first at a frequency of 15 to 30 min/time and 2 to 6 times/d and maintaining a lateral decubitus position on the unaffected side at rest between jumps. Note, the patients were recommended to jump in a single foot on the unaffected side for lower ureteral stones and jumping in a single foot on the affected side for middle ureteral stones. *Stones in the lower calyx*: the patient is positioned with the head up and feet down (inversion position: 45 to 60 degrees between the coronal plane of the body and the bed surface, or the knee-chest position), lightly patting on the waist of the affected side (10 to 30 min/time, 2 to 3 times/d), and maintaining a lateral decubitus position on the unaffected side for 30 min at rest between jumps. *Stones in the bladder*: urinating in the lateral decubitus position and changing to standing urination after most stones are expelled.

Self-management of stone expulsion	Patients are recommended to record urine volume and color, kidney pain, hematuria, and fever. Patients should visit the hospital in time in case of low back pain, fever, urinary frequency and urgency, and dysuria. The expelled stones are collected as much as possible for composition analysis and subsequent diet guidance.

Postoperative follow-up	Reexamination is performed 1 to 2 weeks after surgery until examination shows that the stones have been eliminated. The follow-up is 3 months but is appropriately prolonged in a few patients.

**Table 2:** Comparison of clinical baseline data between the two groups.

Variables	Total (*n* = 104)	Control group (*n* = 51)	Observation group (*n* = 53)	*p*
Age, year, mean ± SD	39.7 ± 10.5	41.0 ± 11.0	38.4 ± 9.9	0.215
Gender, *n* (%)				0.931
Male	73 (70.2)	36 (70.6)	37 (69.8)	
Female	31 (29.8)	15 (29.4)	16 (30.2)	
Size of stones, mean ± SD	49.2 ± 34.9	52.9 ± 38.8	45.7 ± 30.6	0.295
Number of stones, *n* (%)				0.222
1	100 (96.2)	50 (98)	50 (94.3)	
2	3 (2.9)	0 (0)	3 (5.7)	
3	1 (1.0)	1 (2)	0 (0)	
Location of stones, *n* (%)				0.456
Renal calculi	8 (7.7)	4 (7.8)	4 (7.5)	
Distal ureteral calculi	2 (1.9)	0 (0)	2 (3.8)	
Upper ureteral calculi	62 (59.6)	30 (58.8)	32 (60.4)	
Lower ureteral calculi	19 (18.3)	12 (23.5)	7 (13.2)	
Middle ureteral calculi	13 (12.5)	5 (9.8)	8 (15.1)	
Education level, *n* (%)				0.044
Junior and senior high school	70 (67.3)	32 (62.7)	38 (71.7)	
Technical secondary school and junior college	21 (20.2)	15 (29.4)	6 (11.3)	
Undergraduate and above	13 (12.5)	4 (7.8)	9 (17)	
Occupation, *n* (%)				0.002
Students	4 (3.8)	3 (5.9)	1 (1.9)	
Officials	1 (1.0)	1 (2)	0 (0)	
Self-employed people	9 (8.7)	9 (17.6)	0 (0)	
Workers	29 (27.9)	11 (21.6)	18 (34)	
Others	61 (58.7)	27 (52.9)	34 (64.2)	
Number of lithotripsy, *n* (%)				0.258
1	91 (87.5)	47 (92.2)	44 (83)	
2	9 (8.7)	2 (3.9)	7 (13.2)	
3	4 (3.8)	2 (3.9)	2 (3.8)	
Voltage 1, mean ± SD	81.6 ± 7.2	81.8 ± 6.9	81.5 ± 7.6	0.837
Voltage 2, mean ± SD	90.4 ± 10.0	91.1 ± 10.4	89.8 ± 9.8	0.516
Average of voltage, mean ± SD	86.0 ± 8.4	86.4 ± 8.4	85.6 ± 8.4	0.632
Number of shocks, mean ± SD	2250.1 ± 477.7	2356.3 ± 426.9	2147.9 ± 505.0	0.025
Time of stone expulsion, mean ± SD	26.5 ± 16.6	25.8 ± 17.2	27.1 ± 16.1	0.689
Comorbidity, *n* (%)				0.924
0	84 (80.8)	41 (80.4)	43 (81.1)	
1	20 (19.2)	10 (19.6)	10 (18.9)	

Enumeration data were expressed as *n* (%), and chi-square (*χ*^2^) test or Fisher's exact test was used for comparison between groups. Measurement data were expressed as mean ± standard deviation (SD), and *t*-test was used for comparison between two groups.

**Table 3:** Comparison of compliance behavior between the two groups.

Variables	Observation group (*n* = 53)		Control group (*n* = 51)		*χ* ^2^	*P*
	*n*	%	*n*	%		
Complete compliance	41	77.4	23	45.1		
Partial compliance	11	20.6	12	23.5		
Noncompliance	1	1.9	16	31.4	18.310	<0.01

Chi-square (*χ*^2^) test was used for the comparison between groups.

**Table 4:** Comparison of stone expulsion time.

Group	Complete compliance (*n* = 64)	Partial compliance (*n* = 23)	Non-compliance (*n* = 17)
Stone expulsion time (day)	18.5 ± 13.5	26.7 ± 12.7^∗^	30.7 ± 14.9^∗∗^

^∗^ *P* < 0.05 and ^∗∗^*P* < 0.01 vs. complete compliance.

**Table 5:** Comparison of postoperative pain behavior between the two groups.

Variables	Complete compliance (n =64)	Partial compliance (n =23)	Non-compliance (n =17)	*P*
Pain behavior				
Lumbar soreness	31 (48.4%)	10 (43.5%)	11 (64.7%)	0.382
Nausea and vomiting	13 (20.3%)	11 (47.8%)	5 (29.4%)	**0.048**
Frowning	23 (35.9%)	6 (26.1%)	3 (17.6%)	0.299
Lacrimation	7 (10.9%)	6 (26.1%)	8 (47.1%)	**0.005**
Cold sweat	6 (9.4%)	3 (13.0%)	6 (35.3%)	**0.047**

## Data Availability

The data used to support the findings of this study are available from the corresponding author upon request.

## References

[1] Desai M., Sun Y., Buchholz N. (2017). Treatment selection for urolithiasis: percutaneous nephrolithomy, ureteroscopy, shock wave lithotripsy, and active monitoring. *World Journal of Urology*.

[2] Pereira-Arias J. G., Gamarra-Quintanilla M., Urdaneta-Salegui L. F. (2017). Current status of extracorporeal shock wave lithotripsy in urinary lithiasis. *Archivos Españoles de Urología*.

[3] Fan W. L., Wang C. Q., Wang Q., Yang J. K. (2011). Treatment of 886 cases with urinary calculus with ESWL. *Medical Journal of West China*.

[4] Ye Z. Q. (2005). Research status and prospect of urinary calculi. *Chinese Journal of Experimental Surgery*.

[5] Zhou J., Liang C. C., Ye Y. P. (2014). Treatment of severe post-ESWL complications. *Chinese Journal of Urology*.

[6] Zhang Z. W., Lu X. Y. (2017). The optimal treatment timing for extracorporeal shock wave lithotripsy in patients with renal colic. *International Journal of Urology and Nephrology*.

[7] Zhang Z. W., Lu X. Y. (2016). Application of precise health education in patients after ESWL. *Journal of Modern Urology*.

[8] Zhu K., Xin L. I., Wei L. I. (2013). Analysis of factors influencing the efficacy of extracorporeal shock wave lithotripsy in the treatment of ureteral calculus. *Journal of Modern Urology*.

[9] Li N. X., Tang M., Wang Z. J., Ren X. H., Liu D. P. (2001). Study of the behavior of following prescription. *Modern Preventive Medicine*.

[10] Zhang C. Y., Fan X. Y., Jiang K. (2017). Effect of rehabilitation on health education in patients with liver cirrhosis portal hypertension medical behavior. *Chinese Journal of Health Education*.

[11] Nabi G., Baldo O., Cartledge J., Cross W., Joyce A. D., Lloyd S. N. (2003). The impact of the Dornier Compact Delta lithotriptor on the management of primary ureteric calculi. *European Urology*.

[12] Skolarikos A., Alivizatos G., de la Rosette J. (2006). Extracorporeal shock wave lithotripsy 25 years later: complications and their prevention. *European Urology*.

[13] Yue C. (2013). Analysis and countermeasures discussion on non-compliance to medical orders behavior. *Chinese Medical Ethics*.

